This article has been retracted.

# Optimization and Evaluation of an Intelligent Short-Term Blood Glucose Prediction Model Based on Noninvasive Monitoring and Deep Learning Techniques

**DOI:** 10.1155/2022/8956850

**Published:** 2022-04-11

**Authors:** Yongjun Zhang, Guangheng Gao

**Affiliations:** ^1^School of Information Engineering, Shandong Youth University of Political Science, Jinan, China; ^2^Key Laboratory of Intelligent Information Processing and Information Security in Universities of Shandong, Jinan, China; ^3^Biology Institute, Qilu University of Technology(Shandong Academy of Sciences), Key Laboratory for Biosensors of Shandong Province, Jinan, China

## Abstract

Continuous noninvasive blood glucose monitoring and estimation management by using photoplethysmography (PPG) technology always have a series of problems, such as substantial time variability, inaccuracy, and complex nonlinearity. This paper proposes a blood glucose (BG) prediction model for more precise prediction based on BG series decomposition by complete aggregation empirical mode decomposition based on adaptive white noise (CEEMDAN) and the gated recurrent unit (GRU) that is optimized by improved bacterial foraging optimization (IBFO). Hierarchical clustering technology recombines the decomposed BG series according to their sample entropy and the correlations with the original BG trends. Dynamic BG trends are regressed separately for each recombined BG series by the GRU model to realize the more precise estimations, which are optimized by IBFO for its structure and superparameters. Through experiments, the optimized and basic LSTM, RNN, and support vector regression (SVR) are compared to evaluate the performance of the proposed model. The experimental results indicate that the root mean square error (RMSE) and mean absolute percentage error (MAPE) of the 15-min IBFO-GRU prediction is improved on average by about 13.1% and 18.4%, respectively, compared with those of the RNN and LSTM optimized by IBFO. Meanwhile, the proposed model improved the Clarke error grid results by about 2.6% and 5.0% compared with those of the IBFO-LSTM and IBFO-RNN in 30-min prediction and by 4.1% and 6.6% in 15-min ahead forecast, respectively. The evaluation outcomes of our proposed CEEMDAN-IBFO-GRU model have high accuracy and adaptability and can effectively provide early intervention control of the occurrence of hyperglycemic complications.

## 1. Introduction

Diabetes is a hyperglycemia disorder with abnormal glucose metabolism. According to the data from the WHO, there are about 450 million diabetic patients worldwide [1, 2]. By 2045, this figure may reach 700 million. The gradual maturity of continuous glucose monitoring (CGM) technology has dramatically prevented BG-related syndromes in recent years. However, the BG concentration time series includes time-variation, nonlinearity, and instability [3]. It has seriously affected the accuracy of BG level estimation and restricted the closed-loop control performance of the artificial pancreas [4].

At present, the continuous BG trend prediction systems with high and low BG alarm lines to generate timely warnings always have different degrees of deviation [5, 6]. The reason is that the injected insulin takes a particular time to reduce the BG levels. The human body consumes carbohydrates to maintain the normal physiological state by maintaining a reasonable BG level. Therefore, it is necessary to accurately predict BG levels to effectively avoid abnormal BG events in the short period ahead and ensure complementary treatment within the valid time range. If the BG prediction deviates from the actual BG trends, it will lead to a false BG alarm, which will lead to making an approximate amount of insulin injection and cannot alleviate adverse symptoms of abnormal BG changes well, even endangering the safety of patients.

With the development of noninvasive sensing and deep learning techniques, researchers use BG and other data indicators obtained by various sensors to build a data-driven BG prediction model for accurate and timely prediction of abnormal BG trends [7–11]. Alia et al. [12] constructed a blood glucose prediction model based on a neural network and studied the influence of different input characteristics on the prediction accuracy. Support vector regression is used to predict short-term blood glucose, used the differential evolution method to optimize its parameters, and achieved good prediction results [13]. In addition, some scholars have constructed BG prediction models by using ARIMA, the Gaussian mixture model, reinforcement learning, random forests, the Kalman filter, and other methods [10, 14–16]. Liu et al. [17] designed one kind of physique-based fuzzy granular modeling method for BG estimation to achieve a good prediction effect, which took PLS, SVR, random forests, AdaBoost, and the ANN as a comparison algorithm group. Wu et al. [18] proposed the accurate XGBoost-BLR model for type 2 diabetes mellitus prediction in comparison with other existing methods. These models can achieve short-term BG prediction to a certain extent, but when the time step increases, the forecasting effect will be greatly reduced. Therefore, it is necessary to study further to improve the estimation accuracy as much as possible.

Recurrent neural networks (RNNs) have more prominent advantages over other artificial neural network structures in terms of time series modeling. For the actual practice of time series prediction, RNN modeling is similar to auto-regressive analysis, but it can build models much more complex than traditional time series. Basic RNNs and its two variants, long short-term memory (LSTM) and the gated recurrent unit (GRU), have been proved to have a better prediction effect than traditional machine learning methods on time series prediction [1, 8, 19]. When the prediction step increases, its prediction effect is also significantly better than that of traditional methods. Considering the nonlinearity and complexity of the BG series, this paper applies the optimized GRU by the improved bacterial foraging algorithm to the field of BG prediction [19, 20]. The wrist was selected to acquire the pulse signals simultaneously, and body temperature series with minimally invasive extraction of BG signals from upper-arm-based subcutaneous interstitial fluid was selected to construct the training and test dataset [21, 22]. Experimental results show that our proposed method has high accuracy and adaptability and is better than similar types of deep learning methods.

The rest of this paper is organized as follows.  Section 2 presents the background and previous knowledge of noninvasive BG monitoring and its feature extraction issues. The time series decomposition technologies, deep learning models, and BFO optimization algorithms are introduced to improve the prediction performance by utilizing deep learning techniques. In addition, the CEEMDAN-IBFO-GRU model is constructed through the previously sampled BG and PPG dataset. The creation and optimization process of the whole intelligent model is also described in detail in this section. Through experiments, in Section 3, the performance and accuracy of the proposed model are compared with the commonly used machine learning techniques in the actual experiments in BG-forecasting evaluations. Finally, Section 4 concludes this paper and provides possible future applications in clinical fields.

## 2. Materials and Methods

### 2.1. Dynamic Noninvasive and Minimally Invasive BG Monitoring

Photoplethysmography (PPG) is an optical measurement technique that can be used to perform noninvasive BG detection using near-infrared absorption techniques [23–26]. Specific processing of PPG signals can reveal new information about human hemodynamic characteristics and blood composition. In this study, the optical sensor with reflection mode is used to obtain high-quality PPG signals from the subjects' wrists, extract the key PPG parameters (Teager–Kaiser energy, heart rate, spectral entropy, logarithmic features of spectral energy, etc.) and body temperature, and synchronously combine with minimally invasive BG monitoring series to precisely predict the short-term BG trends. PPG signals are sampled with a frequency of 50 Hz and packaged in ATmega328P, which are more reliably harvested using ZigBee technology, and these data are sent to a backend computer using a star-type network structure. Meanwhile, the dynamic BG monitoring data are wirelessly transmitted to a smart phone by Bluetooth once every three minutes. It relies on WiFi to send these data to the backend computer for the training dataset constructions. The BG level prediction modeling process is illustrated in Figure 1.

However, the current photometric-measured signal is more unstable and imprecise, hindering the development of noninvasive BG prediction technologies. The minimally invasive BG monitoring sensors, such as Medtronic, Dexcom, and Abbott, implant the glucose sensor into the subcutaneous tissue through the skin, which dramatically reduces patients' pain and generally shows more accurate monitoring results than noninvasive technologies. Therefore, well-established training and test datasets will provides a reliable source for deep learning models to calibrate and optimize the noninvasive BG prediction modeling process by integrating the synchronous noninvasive PPG data and minimally invasive BG data. The multidimensional feature matrix is extracted as the input of deep learning models according to *S*_window_′(*t*) and *S*_window_^″^(*t*) output by the noninvasive acquisition module. The following feature matrix is used as input data for deep learning techniques. The specific definitions of the PPG features, as well as the body temperature BT, are expressed as equations (1)–(7).

(1) $$\begin{array}{c} X_{i}=\left({\text{KTE}}^{\mu },{\text{KTE}}^{\sigma },{\text{KTE}}^{iqr},{\text{KTE}}^{skw},{\text{HR}}^{\mu },{\text{HR}}^{\sigma },{\text{HR}}^{iqr},{\text{HR}}^{\text{skew}},Hs^{\mu },Hs^{\sigma },Hs^{iqr},Hs^{skew},\;\log\;E^{\delta },\;\log\;E^{iqr},\text{BT}\right). \end{array}$$

#### 2.1.1. Teager–Kaiser Energy Features

The Teager–Kaiser energy characteristic calculation formula is as follows:

(2) $$\begin{array}{c} \text{KTE}\left(t\right)=x{\left(t\right)}^{2}-x\left(t+1\right)x\left(t-1\right). \end{array}$$

Using formula (3), the slice real-time energy value can be obtained:

(3) $$\begin{array}{c} {\text{KTE}}_{n}\left(t\right)=S_{\text{frame}}\left(t,n\right)-S_{\text{frame}}\left(t+1,n\right)S_{\text{frame}}\left(t-1,n\right), \end{array}$$

where *t*  =  1,…, *L*_frame−1_.

The mean value (KTE_*n*_^*μ*^), variance (KTE_*n*_^*σ*^), interquartile spacing (KTE_*n*_^*iqr*^), and slope of a single slice (KTE_*n*_^shew^) can be obtained through KTE_*n*_(*t*).

#### 2.1.2. Heart Rate Features

The heartbeat interval can be obtained by collecting the waveform to obtain the window heart rate mean value HR^*μ*^, variance HR^*σ*^, interquartile spacing HR^*iqr*^, and skewness HR^shew^.

#### 2.1.3. Spectral Entropy Futures

To apply the fast Fourier transform *S*_frame_(*τ*, *n*), the calculation process is as follows:

(4) $$\begin{array}{c} X_{n}\leftarrow \text{FFT}\left(S_{\text{frame}}\left(\tau ,n\right),L_{\text{FFT}}\right), \end{array}$$

where *L*_FFT_  = 512. *X*_*n*_ is regularized by the following equation:

(5) $$\begin{array}{c} P_{X}^{n}\left[k\right]\leftarrow \frac{{\left|X_{n}\left[k\right]\right|}^{2}}{\sum_{j=1}^{L_{\text{FFT}}}\left|X_{n}\right|{\left.j\right\|}^{2}},\;k=1\ldots L_{\text{FFT}}. \end{array}$$

Finally, the entropy *P*_*X*_^*n*^ is calculated according to the following equation:

(6) $$\begin{array}{c} H\leftarrow P\left[k\right]\log\left(P\left[k\right]\right). \end{array}$$

#### 2.1.4. Logarithmic Features of Spectral Energy

According to the logarithmic formula of spectral energy,

(7) $$\begin{array}{c} H\leftarrow P\left[k\right]\text{log}\left(P\left[k\right]\right). \end{array}$$

The logarithmic variance of spectral energy log*E*^*σ*^ and interquartile difference log*E*^*iqr*^ in the window where the slice is located are calculated.

### 2.2. BG Series Decomposition and Recombination Processing

M. A. Colominas proposed complete ensemble empirical mode decomposition with adaptive noise (CEEMDAN) [27, 28]. This method adds adaptive white noise smoothing pulse interference to each decomposition, which can effectively solve the phenomenon of mode aliasing. This method is specifically utilized to regress modeling after signal decomposition in the fields of short-term BG estimations. The specific decomposition and denoising process is defined using steps 1–5.

**Step 1 .**

Add standard normal white noise *x*(*n*) with different amplitudes to the given target signal *x*(*n*), and construct the signal sequence as

(8) $$\begin{array}{c} x^{i}\left(n\right)=x\left(n\right)+\gamma w^{i}\left(n\right)\left(i=1,\ldots ,I\right). \end{array}$$

**Step 2 .**

In the first stage, the empirical mode decomposition (EMD) is used to decompose the target BG signal; the first modal component is obtained, and the mean value is calculated as

(9) $$\begin{array}{c} {\hat{\text{IMF}}}_{1}\left(n\right)=\frac{1}{I}\sum_{i=1}^{I}{\text{IMF}}_{1}^{i}\left(n\right). \end{array}$$

The first stage margin signal is expressed as

(10) $$\begin{array}{c} r_{1}\left(n\right)=x\left(n\right)-{\hat{\text{IMF}}}_{1}\left(n\right). \end{array}$$

**Step 3 .**

*E*_*k*_(·) is defined as the IMF component after the EMD decomposition of signal data. By decomposing the sequence *r*_1_(*n*)+*γ*_1_*E*_1_(*w*^*i*^(*n*)), it can be obtained that the IMF component in the second stage is as follows:

(11) $$\begin{array}{c} {\hat{\text{IMF}}}_{2}\left(n\right)=\frac{1}{I}\sum_{i=1}^{I}E_{1}\left\{r_{1}\left(n\right)+\gamma_{1}E_{1}\left[w^{i}\left(n\right)\right]\right\}. \end{array}$$

**Step 4 .**

By analogy, the *k* − *th* residual component is expressed as

(12) $$\begin{array}{c} r_{k}\left(n\right)=r_{k-1}\left(n\right)-{\hat{\text{IMF}}}_{k}\left(n\right). \end{array}$$

The *k*+1 IMF component is

(13) $$\begin{array}{c} {\hat{\text{MF}}}_{k+1}\left(n\right)=\frac{1}{I}\sum_{i=1}^{I}E_{1}\left\{r_{k}\left(n\right)+\gamma_{k}E_{k}\left[w^{i}\left(n\right)\right]\right\}. \end{array}$$

**Step 5 .**

Repeat step (4) until the remaining components cannot meet the EMD decomposition conditions or the iteration ends. Finally, the target data sequence *x*(*n*) is decomposed into equation (14), where *R*(*n*) is the final residual component.

(14) $$\begin{array}{c} x\left(n\right)=\sum_{k=1}^{K}{\hat{\text{IMF}}}_{k}\left(n\right)+R\left(n\right). \end{array}$$

To study changing features of the BG series, sample entropy can be used to measure the complexity of the time series [29]. It has advantages such as no self-matching problem of approximate entropy and less computation cost. Suppose *X*(*t*) is a sequence with a data length *n*. The series *X*(*t*) is constructed into a new series *Y*(*t*) with *m*−dimension by the following expression:

(15) $$\begin{array}{c} Y\left(i\right)=\left\{y\left(1\right),y\left(2\right),\ldots ,y\left(m-1\right),y\left(m\right)\right\}\\ =\left\{X\left(1\right),X\left(2\right),\ldots ,X\left(N-m\right),X\left(N-m+1\right)\right\}. \end{array}$$

The distance *d*[*y*(*i*), *y*(*j*)] between *y*(*i*) and *y*(*j*) in (16) is the absolute value of the maximum difference between all their elements.

(16) $$\begin{array}{c} d\left[y\left(i\right),y\left(j\right)\right]=\text{max}\left[y\left(i+k\right)-y\left(j+k\right)\right]. \end{array}$$

The sample entropy of the original series *S*(*m*, *r*) is defined as

(17) $$\begin{array}{c} \left\{\begin{array}{c} S\left(m,r\right)=\underset{N⟶+\infty }{\lim}\left\{-\ln\left(\left[\frac{A^{m}\left(r\right)}{B^{m}\left(r\right)}\right]\right)\right\},\\ A^{m}\left(r\right)={\left(N-m+1\right)}^{-1}\cdot \sum_{i=1}^{N-m+1}A_{i}^{m}\left(r\right),B^{m}\left(r\right)={\left(N-m+1\right)}^{-1}\cdot \sum_{i=1}^{N-m+1}B_{i}^{m}\left(r\right), \end{array}\right. \end{array}$$

where *m* represents the embedding dimension of the time series, *r* represents the similarity capacity, and *S*(*m*, *r*) represents the sample entropy of the original series. Thus, *B*^*m*^(*r*) and *A*^*m*^(*r*) are the probabilities of the two-series matching *m* − *th* and (*m*+1) − *th* sampled points, respectively, under the similarity tolerance *r*. Generally, *m* is set to 1 or 2, and *r* selects a value between 0.1 and 0.25.

After the acquisition of the decomposed BG signals, it is reasonable to get the complexity of the BG series by calculating its sample entropy to avoid the problem of large error generation caused by directly applying the deep learning models for estimation training and modeling. Then, according to the correlation between the decomposed and the original BG series, the disintegrated BG series are recombined for more accurate prediction modeling by hierarchical clustering according to its complexities. The specific reconstruction process for BG signals is discussed in Section 3.3.

### 2.3. GRU Prediction Model

Ren [30] et al. proposed an improved recurrent neural network (LSTM) in 1997. The LSTM model uses memory cells to store and output information to solve the gradient explosion problems that easily occur in the RNN model. LSTM has good predictability for long series and is widely used to predict time series data. However, due to its complex internal structure, training of the LSTM network and its superparameters usually takes a long time. Rui [31] proposed a gated recurrent unit neural network (GRU) that is based on LSTM. Compared with LSTM, the training parameters are few, and the prediction effect is close to the LSTM. The structural unit of the GRU neural network is shown in Figure 2.

The GRU′s internal unit is similar to the internal unit of LSTM, except that the GRU combines the forgetting gate and output gate in LSTM into a single update gate. Therefore, there are only updated doors and reset doors in the GRU, and their internal relationship is as follows:

(18) $$\begin{array}{c} R_{t}=\sigma \left(W_{rx}X_{t}+W_{rh}H_{t-1}\right),\\ Z_{t}=\sigma \left(W_{zx}X_{t}+W_{zh}H_{t-1}\right),\\ {\bar{H}}_{t}=\text{tan}h\left(W_{sh}R_{t}H_{t-1}+W_{sx}X_{t}\right),\\ H_{t}=\left(1-Z_{t}\right)H_{t-1}+Z_{t}{\bar{H}}_{t}, \end{array}$$

where *X*_*t*_ is the input vector at time *t*, *R*_*t*_ is the reset gate vector at time *t*, and the gate vector *Z*_*t*_ is updated at *t*. The hidden layer output vector is *H*_*t*_ at time *t*. ${\bar{H}}_{t}$ is the updated candidate vector after the updation. *W*_*sh*_, *W*_*sx*_, *W*_*zx*_, *W*_*zh*_ , *W*_*rx*_, and *W*_*rh*_ are the weight matrices between the connection vectors. *σ* denotes the sigmoid function.

### 2.4. Bacterial Foraging Optimization (BFO)

Bacterial foraging optimization (BFO) is a biologically inspired swarm intelligence optimization algorithm that simulates the foraging behavior of bacteria to obtain maximal energy during the searching process [32, 33]. This algorithm is designed to find the global optimal value and shows better performance than the basic PSO and genetic algorithm. Because the BFO algorithm is easy to jump out of the local minimum, its improved algorithm can accelerate the convergence speed of the algorithm. BFO simulates the behavior of *Escherichia coli* swallowing food in the human intestine and solves the problem by the following simulating behaviors.

#### 2.4.1. Elimination and Dispersal

When the local environment of bacteria changes or mutates gradually (such as food depletion or sudden temperature increase), bacteria will randomly move to a new area with a given probability *P*_*ed*_ to cope with abnormal changes.

#### 2.4.2. Chemotaxis

Bacteria will rotate and swim toward food-rich areas. Rotation refers to pointing in a new direction. The chemotaxis behavior is shown as follows:

(19) $$\begin{array}{c} \theta^{i}\left(j+1,k,l\right)=\theta^{i}\left(j,k,l\right)+C\left(i\right)\frac{\Delta \left(i\right)}{\sqrt{\Delta^{T}\left(i\right)\Delta \left(i\right)}}, \end{array}$$

where *θ*^*i*^(*j*, *k*, *l*) represents the position of bacteria *i* after the trend, *j* − *th* replication, and *l* − *th* dispersion; *C*(*i*) is the trend step of the bacteria, and Δ(*i*) is a unit vector of bacteria in the random direction in the search space.

#### 2.4.3. Swarming

When bacteria forage, there are gravitational and repulsive forces among different individuals. It makes bacteria gather more in some areas with moderate food abundance. The swarming behavior is expressed as

(20) $$\begin{array}{c} J_{cc}\left(\theta ,P\left(j,k,l\right)\right)=\sum_{i=1}^{S}J_{cc}\left(\theta ,\theta^{i}\left(j,k,l\right)\right)\\ =\sum_{i=1}^{S}\left[-d_{\text{attractan }}\text{exp}\left(-w_{\text{attractant}}\sum_{m=1}^{P}{\left(\theta_{m}-\theta_{i}^{m}\right)}^{2}\right)\right]\\ +\sum_{i=1}^{S}\left[-h_{\text{repellant}}\text{exp}\left(-w_{\text{repellant}}\sum_{m=1}^{P}{\left(\theta_{m}-\theta_{i}^{m}\right)}^{2}\right)\right]. \end{array}$$

where *d*_attractant_ is the gravitational depth, *w*_attractant_ is the gravitational width, *h*_repellant_ is the repulsive height, *w*_repellant_ is the repulsive width, *θ*_*i*_^*m*^ is the *m* − th component of bacteria *i*, *θ*_*m*_ is the *m* − th component of all other bacteria, and *P*(*j*, *k*, *l*) is the position of individuals in the population after the *j* − th trend operation, *k* − th replication operation, and *l* − th migration operation.

#### 2.4.4. Reproduction

Bacteria with weak foraging ability will be eliminated, and bacteria with strong foraging ability will replicate. The following equation is called the fitness value of bacteria *i*:

(21) $$\begin{array}{c} J_{\text{health}}^{i}=\sum_{i=1}^{N_{c}}J\left(i,j,k,l\right), \end{array}$$

where *J*(*i*, *j*, *k*, *l*) is the fitness value of the *i* − *th* bacterium after the *j* − *th* trend operation, *k* − *th* replication operation, and *l* − *th* elimination and dispersal. By arranging *J*_health_^*i*^, the algorithm will discard half of the bacteria with larger fitness and copy the other half of the bacteria with smaller fitness.

In the process of BG estimation optimization, bacteria present a solution; the location of the bacterium in the search space corresponds to the solution of the optimization problem, and the fitness value of the optimization function, that is, the value of the objective function, represents the excellence of the superparameter selection for deep learning prediction modeling.

### 2.5. The Intelligent BG Prediction Modeling

To improve the training and tuning effect of the GRU prediction model, structure and superparameters should be reasonably selected and adjusted. Theoretically, the complexity of the network increases with the increase in the number of hidden layers and the number of neurons in the hidden layer. Meanwhile, such complexities and computation costs of deep learning networks are also increased dramatically. Therefore, scientific and reasonable optimization of models' superparameters such as the learning rate and maximum iteration times can reduce the complexity of the model to a certain extent and also improve the convergence speed as well as the prediction accuracy. The improved bacterial foraging algorithm (IBFO) that has characteristics such as good convergence performance and high optimization accuracy, which is designed in this study, learns from ideas of particle swarm optimization (PSO) [34]. It trains and optimizes the structure and superparameters of the GRU neural network according to the existing PPG and BG series to train and construct a short-term BG level prediction model with higher prediction accuracy.

In a traditional BFO algorithm, however, the invariance of step size will affect the accuracy of the optimal solution, and the invariance of elimination and dispersal probability will slow down the convergence speed in the later stage of the algorithm. In consideration of such shortcomings, the following improvements are proposed to improve the performance of the basic BFO.

The improved BFO will dynamically adjust its step size to improve the optimization accuracy. The basic rule for improvement of the convergence speed is to increase the foraging step size when the distance between the two individuals is far, and vice versa. The following equation can achieve the adaptive adjustment for foraging step size:
  (22) $$\begin{array}{c} C{\left(i\right)}^{\prime }=\lambda \left(\frac{C_{\text{max}}}{j\times k\times l}\right)\frac{J_{i}}{J_{\text{max}}}, \end{array}$$
where *J*_*i*_ is the fitness value of the current bacteria *i*, *J*_max_ is the maximum fitness value of all current bacteria, *C*_max_ is a quarter of the sum of the maximum and minimum value of the d-dimensional optimization range, *j*, *k*, and *l* are the current trend, replication, and elimination and dispersal times, respectively, and *λ* is a random number between 0 and 1.
Learning from the idea of the learning factor of particle swarm optimization, the swimming of a bacterium is not only limited by its foraging ability but also affected by other bacteria [35]. That is to say, a bacterium's fitness function value is compared with that of the current bacteria with the best foraging ability, and its foraging ability is improved by communicating with and learning from the bacteria with better foraging ability. Its function is given by
  (23) $$\begin{array}{c} \Delta {\left(i\right)}^{\prime }=\Delta \left(i\right)+\lambda C_{1}\left(J_{\text{max}}-J_{i}\right)+\lambda C_{2}\left({\bar{J}}_{\text{global}}-J_{i}\right), \end{array}$$
where Δ(*i*) is a unit vector of bacteria in the random direction in the search space, *C*_1_ and *C*_2_ are learning factors, and ${\bar{J}}_{\text{global}}$ is the average fitness of all bacteria at that moment.
Finally, an adaptive elimination and dispersal probability of IBFO is designed to solve the drawbacks of less flexibility of the fixed migration. All bacteria migrate to a new region with fixed *P*_*ed*_, which may lead to the loss of elite individuals and the reduction in convergence speed, accuracy, and stability of the algorithm. The improvement is realized by the following formula:
  (24) $$\begin{array}{c} P_{ed}^{\prime }\left(i\right)=\left[\frac{\left(J_{\text{max}}-J_{i}\right)}{\left(J_{\text{max}}-J_{\text{min}}\right)}\right]\times p_{ed}, \end{array}$$
where *J*_max_ and *J*_min_ are the maximum and minimum fitness values of all bacteria at present and *P*_*e*  *d*_ and *P*_*ed*_′(*i*) are the fixed and adaptive elimination and dispersal probability, respectively.
Through the improvement, the bacterial migration probability with a small fitness function value is increased. This will ensure that the bacteria with the best foraging ability will be migrated to improve the stability of the algorithm. The specific algorithm for the noninvasive intelligent BG prediction modeling and evaluation is described in the following three parts, and the specific procedures are illustrated in Figure 3.
Part 1. The BG and related signal acquisition, decomposition, and recombination. The training and the test dataset are constructed by obtaining the PPG features, body temperature, and continuous real BG series simultaneously. Then, the BG signal is decomposed by CEEMDAN, and its sample entropy is also calculated to get the complexities of each decomposed signal. Afterward, the disintegrated signal is recombined into high-, medium-, and low-correlation series by hierarchical clustering. These rearranged series are proved to be more suitable for deep learning models to regress in each component and implement more accurate forecasting by reconstructing each regrouped estimation results.
Part 2. The optimization of superparameters of the prediction model. To initialize the parameters of the improved BFO algorithm, the number of output layer and input layer nodes, hidden layers, and learning rate of the GRU neural network are determined according to the original series and actual objectives. The improved BFO will dynamically adjust its step size and improve the foraging ability with adaptive migration probability to provide more optimized superparameters for the GRU model.
Part 3. The BG trend prediction and its performance evaluation. The recombined BG signals are regressed by the IBFO-optimized GRU model and to reconstruct the final estimated BG results. Consequently, the series are denormalized to get the real BG trends. Finally, the CEEMDAN-IBFO-GRU model is evaluated by MAPE, RMSE, and the Clarke error grid criterion and compared with other machine learning methods.

## 3. Results and Discussion

The experimental environment of this paper is Windows 10 operating system. Python 3.10 and the machine learning framework PyTorch 1.1 are used for deep learning modeling and testing. The hardware configuration is a 64-bit operating system, and the processor is Intel(R) Core (TM) i7-4900MQ CPU 2.80 GHz with 16GB RAM.

### 3.1. Data Source Preparation and Preprocessing

In this research, the dynamic noninvasive BG monitoring device that is worn on the wrist of patients dynamically measures BG levels by using an optical PPG acquisition module (MKB0805, YUNKEAR Ltd., Shenzhen, China). Meanwhile, the minimally invasive CGM (YUWELL Ltd., China) synchronously collects more accurate GB trends to support the construction of calibration datasets, which are collected by dynamic BG records in the Shandong rehabilitation research center, China. The real continuous BG data of 12 patients were investigated. The BG levels of diabetic patients are continuously and dynamically monitored and recorded at an interval of three minutes, and the trends are monitored for three days (about 72 hours), with a total of 1440 sampling points in our experiment, excluding the points with breakpoints, discontinuities, and serious interference during the monitoring. The sampled BG series of each patient is obtained and divided into a training dataset and test dataset, which accounts for 70% and 30%, respectively. Sliding windows and single-step prediction are used for the BG dynamic estimation processes. The acquired PPG features in the last 3 hours are utilized for GB level estimation in 15- or 30-minutes. The specific dataset construction for the intelligent BG estimation modeling is shown in Figure 4.

Due to the different dimensions between sampled feature data, in this study, the max-min standardization method is used for time series normalization as follows:

(25) $$\begin{array}{c} x_{\text{Normalization}}=\frac{x-\text{Min}\left(x\right)}{\text{Max}\left(x\right)-\text{Min}\left(x\right)}, \end{array}$$

where Max(*x*) and Min(*x*) denote the maximum and the minimum value of BG series, respectively.

### 3.2. Model Performance Evaluation Criterion

To quantify the prediction performance of the proposed models, root mean square error (RMSE), mean absolute percentage error (MAPE), and Clarke error grid analysis (EGA) are selected as the performance measurements for the model evaluation. The calculation of RMSE and MAPE is as follows:

(26) $$\begin{array}{c} \text{RMSE}=\sqrt{\frac{1}{n}\sum_{i=1}^{n}{\left(x_{i}-\bar{x_{i}}\right)}^{2}}. \end{array}$$

The average absolute percentage error is calculated as follows:

(27) $$\begin{array}{c} \text{MAPE}=\frac{1}{n}\sum_{i=1}^{n}\left|\frac{x_{i}-{\bar{x}}_{i}}{x_{i}}\right|\times 100. \end{array}$$

Here, *n* is the number of samples, *x*_*i*_ is the actual value of the *i* − *th* sample, and $\bar{x_{i}}$ is the predicted value of the *i* − *th* sample.

Clarke error grid analysis was developed to evaluate the clinical accuracy of measured BG and standard reference BG data. This method can evaluate the clinical effect difference between the actual BG level and the predicted level. This method uses the Cartesian diagram principle to evaluate the accuracy of the BG prediction methods according to the probability that the predicted values fall in areas A, B, C, D, and E.

### 3.3. The Experimental Results

The minimally invasive BG signal is decomposed by CEEMDAN for training and modeling as shown in Figure 5, and it disassembles the intrinsic mode function (IMF) from IMF1 to IMF7 and the residuals.

According to the complexity of the decomposed signal group, the sample entropy is calculated, and the similarity is calculated by hierarchical clustering. Through clustering calculation, the signals are classified as high, medium, and low complexity (*H*_*t*_, *M*_*t*_, and *L*_*t*_) in clusters 1 to 3. The complexity of the decomposed BG series is regrouped according to the correlation with the original BG series. The clustering process of recombined signals and its correlation with the original BG series is demonstrated in Figure 6.

The decomposed signals are clustered and reconstructed according to their complexities, and the specific combinations are demonstrated in Table 1. The Pearson correlation coefficient is used to measure how similar the rearranged GB signals and the original BG signals are. To enforce the learning and estimation results of the deep learning modeling construction, the recombined data should be more similar to the originally acquired BG series. The original BG series are reconstructed in high, medium, and low correlations, which will improve the training and estimation performance for the deep learning forecasting models.

The data series of the extracted PPG features are listed in Table 2 as a fundamental training data set for deep learning technique-based BG estimation. The values of the extracted features are normalized in order to facilitate the construction of the training data. In this case, the BG level and its corresponding PPG features are listed to support the BG estimation experiments.

After completing the decomposition of continuous BG series, the improved BFO algorithm is used to tune the deep learning models' hyperparameters. The improved BFO is initialized by the following parameters in detail. The search dimension is *d*=4. The number of bacterial populations *S*, elimination and dispersal behaviors *N*_*ed*_, and chemotaxis behaviors *N*_*c*_ are 50, 2, and 25, respectively. The maximum step of unidirectional motion in the trend behavior *N*_s_ is set to 4. The number of times of the copied behavior *N*_*re*_ is set to 4. The elimination and dispersal probability *P*_*e*  *d*_ is 0.25. The gravitational depth and width are 0.5. In addition, the repulsion depth and width are both 0.5. The local and global learning factors *C*_1_ and *C*_2_ are set to 2.  Figure 7 demonstrates the number of iterations in the training process of IBFO-optimized models (IBFO-RNN, IBFO-LSTM, and IBFO-GRU). Through the training experiments, the number of hidden layer neurons, hidden size, learning rate, and iterations are gradually converged to the optimal value with the update of the algorithm. As can be seen from Figure 7, the number of iterations finally converges to 65, 79, and 95 in IBFO-optimized RNN, LSTM, and GRU, respectively.

Through the training process, we have obtained the optimal combination of parameters with the best performance to modify the model structure and configurations. The number of input and output layers is configured to one for the optimized deep learning models. The loss function is adopted by MSE, and the Adam technology is adopted as the optimizer. The optimized model's structure and its superparameters are described in Table 3.

### 3.4. Model Performance Evaluation and Discussion

This study constructed a short-term BG prediction model based on the CEEMDAN-IBFO-GRU. The whole results of 15- and 30- minute estimation are illustrated in Figure 8 and Figure 9, respectively. S1, S2, and S3 are the zoomed-in pictures in different time segments that indicate the BG estimation trends by using different machine learning methods. It can be seen that the prediction error becomes larger with the increase in prediction step size. In addition, the prediction errors of different patients may have different trends due to the different glycemic fluctuations in patients. Therefore, the BG dynamic trends and its estimation fittings are the average results with similar BMI and health levels. Among them, the best prediction effect of IBFO-GRU is in the forthcoming BG concentration 15 minutes ahead of time; its RMSE is 0.38, and the MAPE is about 6.43%. The prediction RMSE and MAPE increase obviously when the step of BG level estimation in 30-min estimation by using the IBFO-optimized GRU is increased to 0.417 and 7.82%, respectively.

To explore the prediction performance of the proposed intelligent BG prediction method, in this study, it is compared with basic deep learning models RNN, LSTM, GRU, and the support vector regression (SVR, C: 100.0; gamma: 0.01; Kernel function: RBF), and their optimized methods are measured by MAPE and RSME evaluation criteria.  Figure 10 illustrates that the RMSE of IBFO-GRU has improved on average in 15-min prediction by about 3.58% and by 6.29% more than IBFO-LSTM and IBFO-RNN, respectively. In addition, the RMSE improvement is about 13.1% and 16.3% compared that of with PSO- and BFO-based GRU or LSTM. Meanwhile, the MAPE error of IBFO-GRU is increased by about 12.4%, and 18.9% more than that of IBFO-LSTM and IBFO-RNN, respectively. The effect of the CEEMDAN-IBFO-GRU-based BG estimation process has been greatly optimized and improved compared with that of other machine learning techniques.

Finally, to analyze the prediction effect more comprehensively, the Clarke error grid analysis method is purposefully utilized to evaluate the experimental results. The accuracy of the BG estimation models was evaluated by comparing the relationship between the predicted and actual BG concentration. The results are all located in areas A and B, indicating that the results of the analysis are acceptable in theory, that is, the predicted value of the BG level has acceptable detection accuracy in guiding clinical application. Clarke grid errors of the optimized deep learning models in 15 min predictions are shown in Figure 11.

The 15-min ahead BG predicting results are all located in area A, which were predicted by using our proposed method counts as about 98.4%, which are increased by about 4.1% and 6.6% compared to that using IBFO-LSTM and IBFO-RNN, respectively. The prediction results and accuracy of BFO- and PSO-optimized GRU, LSTM, and RNN are similar when applying the dynamic BG level estimation algorithms.  Figure 12 shows that the Clarke error grid results in area A of CEEMDAN-IBFO-GRU with 30-min ahead prediction are improved by about 2.7% and 5.4% when compared with those of other IBFO-optimized LSTM and RNNs and is also increased on average by about 5.4% and 6.2% compared with that of PSO- and BFO-based GRU or LSTM models, respectively. These regions quantify the accuracy of the BG reference values compared to the predicted values for different types of errors.

## 4. Conclusions

This research proposed an intelligent BG level prediction model (CEEMDAN-IBFO-GRU) that is well suitable for the strong time variability and complex nonlinearity of the dynamic BG changes and implements more precise BG forecasting management within short time periods. In this paper, the BG level in human subcutaneous interstitial fluid is continuously monitored through minimally invasive monitoring, and the characteristic sequence based on the PPG signal is synchronously obtained to jointly provide a better training and test dataset for the deep learning algorithm to realize noninvasive continuous BG prediction and early-warning management. BG series is decomposed by CEEMDAN and sample-entropy-based recombination by hierarchical clustering. After that, the recombined BG signals are regrouped according to their correlation with the original signals, which are regressed by the deep learning models to realize a more accurate BG estimation. Furthermore, the improved BFO algorithm is designed for increasing the performance of the deep learning models by optimizing their structures and superparameters. Through experiments, the number of training iterations is fewer, and the structures, as well as the superparameters, are also simple and reasonable for practical BG estimation application in a relatively simple hardware environment. According to the error evaluation criteria RMSE, MAPE, and Clarke error grid analysis, compared with the basic deep learning models LSTM, GRU, and RNN, the results show that the prediction accuracy of CEEMDAN-IBFO-GRU is higher than that of the nonoptimized machine learning methods. Therefore, the proposed noninvasive BG prediction model based on deep learning techniques has been proved to show good performance with relatively high accuracy. In future research, more physiological and activity characteristics should be combined to further improve the blood glucose prediction accuracy for practical clinical application.

## Figures and Tables

**Figure 1:** Overview of the BG concentration prediction modeling.

**Figure 2:** GRU network computing structure.

**Figure 3:** The process of noninvasive BG prediction and evaluation by using the CEEMDAN-IBFO-GRU model.

**Figure 4:** The specific dataset construction for BG estimation modeling.

**Figure 5:** The BG series decomposition by CEEMDAN.

**Figure 6:** The recombination of decomposed BG signals and the correlation with the original BG series.

**Figure 7:** The number of iterations in the IBFO-based deep learning model training process.

**Figure 8:** The short-term BG estimation results in 15 minutes.

**Figure 9:** The short-term BG estimation results in 30 minutes.

**Figure 10:** The short-time BG prediction errors in 15- and 30-minutes.

**Figure 11:** Clarke grid errors of the optimized deep learning models with CEEMDAN in 15 min prediction. (a) IBFO-GRU: area A: 98.4% and B: 1.6%. (b) IBFO-LSTM: area A: 94.3% and B: 5.7%. (c) IBFO-RNN: area A: 91.8% and B: 8.2%. (d) IBFO-GRU: area A: 92.7% and B: 7.3%. (e) IBFO-LSTM: area A: 91.3% and B: 8.7%. (f) IBFO-RNN: area A: 90.1% and B: 9.9%. (g) IBFO-GRU: area A: 92.5% and B: 7.5%. (h) IBFO-LSTM: area A: 91.8% and B: 8.2%. (i) IBFO-RNN: area A: 90.3% and B: 9.7%.

**Figure 12:** Clarke grid errors of the optimized deep learning models with CEEMDAN in 30 min prediction. (a) IBFO-GRU: area A: 96.2% and B: 3.8%. (b) IBFO-LSTM: area A: 93.6% and B: 6.4%. (c) IBFO-RNN: area A: 91.2% and B: 8.8%. (d) IBFO-GRU: area A: 91.3% and B: 8.7%. (e) IBFO-LSTM: area A: 90.9% and B: 9.1%. (f) IBFO-RNN: area A: 88.6% and B: 11.4%. (g) IBFO-GRU: area A: 91.8% and B: 8.2%. (h) IBFO-LSTM: area A: 90.2% and B: 9.8%. (i) IBFO-RNN: area A: 89.6% and B: 10.4%.

**Table 1:** The decomposed BG series and the correlation for reconstruction.

Clustering result	The correlation coefficient with the original BG series	Simple entropy	Decomposed signals
High complexity (*H*_*t*_)	0.143, low correlation	19.121	IMF1

Medium complexity (*M*_*t*_)	0.443, medium correlation	7.094	Res
		6.467	IMF2
		6.681	IMF3

Low complexity (*L*_*t*_)	0.897, high correlation	5.654	IMF4
		5.157	IMF5
		5.021	IMF6
		4.553	IMF7

**Table 2:** The PPG features within a sampling interval.

BG level (mmol/L)	*KTE* ^*μ*^	*KTE* ^*σ*^	*HR* ^*μ*^	*HR* ^*σ*^	…	*HR* ^*iqr*^	*HR* ^*shew* ^
8.9	0.804	0.615	0.861	0.725	…	0.827	0.597
8.2	0.752	0.623	0.843	0.716	…	0.801	0.571
…	…	…	…	…	…	…	…
7.4	0.644	0.578	0.832	0.703		0.793	0.512

**Table 3:** The optimized model's structure and its superparameters by using IBFO.

Models	Parameters	Values
IBFO-GRU	Number of hidden layer neurons	4
	Hidden size	4
	Learning rate	0.0038
	Number of iterations	95

IBFO-LSTM	Hidden size	3
	Number of hidden layer neurons	2
	Learning rate	0.0042
	Number of iterations	79

IBFO-RNN	Number of hidden layer neurons	4
	Hidden size	3
	Learning rate	0.0001
	Number of iterations	65

## Data Availability

The data used to support the findings of this study are included within the article.
